RETRACTED

# Different Grades of Collateral Circulation for Evaluating Cerebral Hemodynamic Status in Carotid Artery Stenosis

**DOI:** 10.1155/2022/8484977

**Published:** 2022-02-02

**Authors:** Weijian Fan, Weihao Shi, Jianjie Rong, Wencheng Guo, Shuangshuang Lu, Jinyun Tan, Bo Yu

**Affiliations:** ^1^Department of Vascular Surgery, Shanghai Pudong Hospital, Fudan University Pudong Medical Center, Shanghai, China; ^2^Department of Vascular Surgery, Huashan Hospital of Fudan University, Shanghai, China; ^3^Department of Vascular Surgery, Suzhou TCM Hospital Affiliated to Nanjing University of Chinese Medicine, Suzhou, China; ^4^Department of Radiology, Huashan Hospital of Fudan University, Shanghai, China

## Abstract

Normally, ipsilateral hemodynamic compromise of patients with carotid stenosis (CS) is subjectively identified by collateral circulation through cerebral angiography in the clinical process. It is unclear whether collaterals would linearly determine cerebral perfusion in CS patients. This study aimed to investigate the independent role of collateral circulation on cerebral perfusion in CS patients and the underlying interrelations among them. From 2017 to 2020, 124 CS patients who underwent carotid endarterectomy (CEA) with both preoperative CTP and digital substruction angiography (DSA) images were enrolled. Division of subgroups was based on degree of CS (50–70%, 70–90%, and near-occlusion (NO)) and grades of collateral circulation by DSA. Differences in CTP parameters between CS patients with different collateral circulation were analyzed. Among 124 CS patients, grades 2 and 3 were highly associated with carotid NO (*n* = 22, 32.35% and *n* = 22, 32.35%) compared with others (*P* < 0.0001). The collateral circulation was found to have poor relation with cerebral perfusion parameters in all enrolled patients but significantly improved ipsilateral cerebral perfusion in patients with carotid NO (*P* < 0.05). Linear hemodynamic compromise was barely related to degree of CS in lobes supplied by middle cerebral artery (MCA) except the frontal lobe (*P* < 0.05). The grades of collateral circulation are positively associated with degree of CS while having nonsignificant effect on cerebral perfusion. Overall, severity of CS is poorly related to hemodynamic status while the perfectibility of compensation defined by grades of collateral circulation effectively alleviates ipsilateral cerebral perfusion deficit in carotid NO.

## 1. Introduction

Atherosclerotic disease occurs frequently at the bifurcation of common carotid artery (CCA), which leads to 15% to 20% of ischemic strokes [1]. According to the results from large, randomized trials, carotid endarterectomy (CEA) has become the accepted standard treatment of choice for patients with carotid stenosis (CS). Besides, as an effective carotid revascularization method, CEA has been testified benefit for symptomatic patients with 50–69% of CS or even greater [2, 3]. Although in patients with stenosis of the internal carotid artery (ICA), the cause of stroke is primarily thromboembolic, the presence of low regional cerebral blood flow is also recognized as an additional risk factor [4]. However, the current threshold for intervention is primarily based on anatomical identification of luminal stenosis and related symptoms, without taking into account compensatory mechanisms, presence of collateral circulation [5], and downstream perfusion status [6], which thus may be insufficient and misleading.

RETRACTED

Several studies have suggested that this risk is further increased if ipsilateral cerebral perfusion is compromised [7, 8], or if cerebral collateral pathways are impaired [9, 10]. The annual stroke risk in symptomatic patients is about 5% but increases up to 40% in patients with severe impairment of cerebral hemodynamics [11]. By the same token, cerebral collateral circulation has long been reported to collectively mitigate the impact of stenosis-induced flow restriction and alter the risk of stroke around the CEA procedure [12, 13]. However, it is still uncertain that to what extent of collateral circulation would be deemed as sufficient ipsilateral cerebral perfusion in CS patients.

CT perfusion (CTP) is introduced to rapidly and easily evaluate cerebral perfusion in patients presenting with underlying hypoperfusion or acute stroke symptoms [14, 15]. Moreover, digital substruction angiography (DSA) is performed as golden standard to evaluate the carotid stenosis and collateral pathways. Previous studies have revealed the correlation between CTP and collaterals in internal carotid artery occlusion (ICAO), while it is still lack of strong evidence for CS patients [16, 17].

The aim of the present study is to first, evaluate the relationship between collateral patterns and the hemodynamic status of CS patients; second, investigate the ipsilateral hemodynamic compromise in subgroups divided by degree of stenosis and interrelation with collateral circulation. By doing so, much more accurate assessment through collateral circulation could provide additional risk stratification for CS patients before revascularization.

## 2. Materials and Methods

### 2.1. Patients and Study Design

All patients provided written consent for the study protocol that was approved by the research and ethics committee in Huashan Hospital of Fudan University. We retrospectively reviewed 359 CS patients who were undertaken CEA operation between January 2017 and September 2020 and 124 of these patients were enrolled combining with both preoperative CTP and DSA images. The exclusion criteria were medical or logistical barriers to performing CTP and/or DSA (*n* = 26), insufficient preoperative CTP and/or DSA (*n* = 175), or refusal (*n* = 34). All patients enrolled were examined and reviewed for demographic characteristics, comorbidities, clinical symptoms, stroke risk factors, and medications by neurologists.

RETRACTED

### 2.2. DSA Protocol and Data Analysis

Patients who were enrolled in the study underwent comprehensive DSA studies with a standard, clinically routine protocol, including injection of both common carotid and vertebral arteries [18]. Carotid and cerebral angiography was administered through the Power injector (Liebel-Flarsheim Angiomat; Illumena, San Diego, California, USA) with 10–12 mL of 60% diluted contrast medium within 1.0 s. Images of angiography were recorded under 7.5 frames/s and were further evaluated by two neurologists. The identification of stenosis was based on the North American Symptomatic Carotid Endarterectomy Trial (NASCET) criteria [2]. Patients were divided into three groups relying on the degree of carotid stenosis (50–70%; 70–90%; and near-occlusion). The diagnosis of carotid near-occlusion (NO), which met the criteria established previously, was made by reviewing catheter angiography imaging [19]. Specifically, consistent with previous illustrative cases, carotid NO was defined as obviously reduced diameter of the ICA with or without full collapse and delayed filling distally [20].

### 2.3. Collateral Circulation

The classification of collateral circulation was consistent with previous studies [10, 21]. Specifically, the biplane intracranial views of selective angiography were examined to assess collateral circulation which was identified by the cross-filling of the ipsilateral territory through contralateral CCA or vertebral artery (VA) injection. The collateral circulation was categorized into 3 grades. Specifically, grade 1 indicates no or slight collateral distribution, often with dilution. Grade 2 indicates small but definite collateral supply and grade 3 indicates near complete collateral with cross-filling of the ipsilateral middle cerebral artery (MCA) after contralateral carotid injection, as shown in Figure 1.

### 2.4. CT Perfusion

As previous studies revealed, CTP scans were performed with the 64-slice detector CT scanner (Philips, Best, the Netherlands) and followed with injection of diluted nonionic contrast material. CTP data were then transferred to a postprocessing workstation (Extended Brilliance Workstation v 3.0, Philips Medical Systems) [22]. Cerebral blood volume (CBV), cerebral blood flow (CBF), mean transit time (MTT), and time to peak (TTP) were calculated using a deconvolution operation (Extend Brilliance Workstation v 3.0, Philips Medical Systems, USA). Absolute values of CTP parameters are subject to the area of regions of interest (ROIs) and are influenced by physiologic factors such as blood pressure [23, 24]. Hence, we used the ratio of the values measured in the ipsilateral hemisphere to those in the contralateral hemisphere for CBV, CBF, MTT, and TTP (rCBV, rCBF, rMTT, and rTTP). Four absolute values obtained from 4 consecutive layers of a given territory were averaged to obtain the mean of CBV, CBF, MTT, and TTP in both ipsilateral and contralateral side. ROIs in both hemispheres including frontal lobe, occipital lobe, temporal lobe, and basal ganglia were manually outlined according to the maps of Damasio [25].

RETRACTED

### 2.5. Statistical Analysis

All analyses were performed using SPSS v.22 software (IBM, Chicago, Illinois, USA). The mean value, standard deviation, and percentage was used, as appropriate, to record demographic characteristics, comorbidities, degree of CS, and collateral circulation. The independent one-way ANOVA test was used to compare the relative CTP parameters in patients with various patterns of collateral circulation or with different degree of stenosis. The Mann–Whitney test was used to compare differences between collateral circulation and cerebral CTP parameters in subgroup of carotid NO patients. Chi-square analysis was performed to investigate the correlation between collateral circulation grades and stenosis degree. Values were expressed as mean ± SD and the significance level was set at *P* < 0.05 for all statistical tests.

## 3. Results

### 3.1. Baseline Characteristics

During the study period, 124 patients with carotid stenosis were recruited (Table 1, mean age, 68.26 ± 8.36 y) and 82.25% of them were male (*n* = 102, 82.25%). The side of carotid stenosis showed no deviation among enrolled patients (Left, *n* = 68, 54.84%) while previous stroke was only found in 18 ones (14.52%). Antiplatelet therapy was prevalent in CS patients (*n* = 107, 86.29%) and 10 patients underwent anticoagulation therapy because of atrial fibrillation. Patients were categorized by the degree of CS while most of them were carotid NO (*n* = 68, 54.84%). The clinical comorbidities of patients such as hypertension, diabetes, hyperlipidemia, smoking, and ischemic heart disease were recorded. Depending on collateral circulation, patients were classified by grade 1 to 3 while grade 1 was noticed for higher proportion (*n* = 74, 59.68%).

RETRACTED

### 3.2. Nonsignificant Relevance between Cerebral CTP Parameters and Collateral Circulation

To evaluate the effect of collateral circulation on ipsilateral hemodynamic status, we then analyzed the correlation between the CTP parameters and collateral grades among all CS patients. The perfusion values were calculated and collected from four ROIs. As shown in Table 2, the rCBV in patients with grade 1 collateral circulation was not significantly different from that in patients with other two patterns. Specifically, nonsignificance revealed by the one-way ANOVA test was found in all ROIs (frontal, *P*=0.926; basal ganglia, *P*=0.996; temporal, *P*=0.533; and occipital, *P*=0.381) and multiple comparison showed no significance between each two groups as well. Besides, rCBF, rMTT, and rTTP still revealed nonsignificance in the corresponding ROIs among all patients with different collateral circulation grades. Interestingly, despite that no significance was found in rMTT and rTTP among patients with different collateral circulation, the grade 3 group which represented intact circle of Willis (CoW) showed decreased rMTT and rTTP in ROIs suggesting that the MTT and TTP in ipsilateral hemisphere were not highly prolonged due to the cerebral autoregulation mechanism and the perfusion balance were maintained.

### 3.3. Complete Collateral Circulation Was Highly Associated with Severe CS

We sought to figure out the relationship between collateral grades and the degree of stenosis in CS patients. Hence, according to previous studies, all patients enrolled were categorized into three groups (50–70%, 70–90%, and NO) depending on the degree of carotid stenosis based on DSA images [26]. As exhibited in Table 3, grade 1 collateral circulation was highly associated with 50–70% and 70–90% of CS, respectively (*n* = 19, 90.48%; *n* = 25, 71.43%), while grade 2 and grade 3 were noted in a low proportion (*n* = 2, 9.52%; *n* = 10, 28.57%). Inversely, patients with carotid NO showed higher percentage of grade 2 and grade 3 (*n* = 22, 32.35%; *n* = 22, 32.35%, *P* < 0.0001^*∗*^) compared with other two groups, indicating that ipsilateral hemisphere with severe CS might have intracranial pressure deficit which would be the driving force for the presence of CoW and compensatory blood flow from contralateral side, as shown in Figure 2.

### 3.4. Cerebral Perfusion Was Poorly Related to Degree of CS except for the Frontal Lobe

To determine the relationship between degree of CS and cerebral perfusion which still failed to reach a consensus according to several studies [17, 27], we further made multiple comparisons between each group. The initial results showed that no significance was found between the degree of stenosis and rMTT in both basal ganglia and temporal lobe (*P*=0.255; *P*=0.331). Still, the same trend was found in rTTP (*P*=0.065; *P*=0.158), indicating that cerebral hemodynamic status had poor correlation with degree of CS in MCA territory of the afflicted hemisphere, as shown in Table 4. Yet, significant elevated rMTT and rTTP were noted in the frontal lobe (*P*=0.037^*∗*^; *P*=0.026^*∗*^) showing a statistically relationship between insufficient perfusion and increasing severity of carotid stenosis. Altogether, cerebral perfusion of frontal lobe was much more sensitive to the change of luminal stenosis while significant functional lobes were less vulnerable owing to cerebral autoregulation and blood flow redistribution.

RETRACTED

### 3.5. Collateral Circulation Had Significant Correlation with Cerebral Perfusion in Patients with Carotid NO

Our study showed nonsignificant relevance between cerebral CTP parameters and collateral circulation grades in all enrolled patients while carotid NO was found highly associated with grade 3 collateral circulation. Thus, in order to identify their internal relationship, we subdivided patients with carotid NO into three groups depending on collateral circulation grades and all these patients were unilateral CS, as shown in Table 5. Slight fluctuation of rCBF value was found in patients with grade 1, 2, and 3 collateral circulations while nonsignificance was reached in selected ROIs (*P*=0.349, *P*=0.322, *P*=0.449). Also, the similar trend was found in both rMTT and rTTP in the frontal lobe (*P*=0.729, *P*=0.917). Nonetheless, except for the frontal lobe which is mostly supplied by anterior cerebral artery (ACA), both basal ganglia and temporal lobe of enrolled patients with grade 3 collateral circulation showed significant reduction in rTTP values (*P*=0.040^*∗*^; *P*=0.047^*∗*^). Besides, significant decline of rMTT was found in basal ganglia in subgroup of grade 3 (*P*=0.024^*∗*^). Collectively, in patients with carotid NO, complete collateral circulation played a pivotal role in relieving ipsilateral cerebral perfusion deficit.

## 4. Discussion

Carotid artery steno-occlusive diseases have been reported to correlate with cerebral hypoperfusion and further lead to cognitive and mobility dysfunction and progression to dementia as results [28]. Several studies have suggested that CS patients with ipsilateral cerebral hemodynamic compromise have impaired cerebrovascular reactivity and aggravate the risk of subsequent transient ischemic attack (TIA) and stroke as compared to those with normal hemodynamics [7, 29, 30]. Furthermore, Schimrigk [31] has shown that the risk of recurrent stroke decreased if more collaterals are recruited. Although cerebral perfusion and collaterals recruitment are crucial and integral to current treatment and stroke prevention paradigms, most consensus recommendations do not include assessments of cerebral hemodynamics in their management algorithms and arbitrarily focus on degree of stenosis and CoW opening based on DSA or CT angiography (CTA) images.

RETRACTED

In our study, CTP was utilized to quantify cerebral perfusion. Hitherto, multiple measurements including single-photon emission tomography, MRI, and 2D/3D arterial spin labeling (ASL) have been developed to assess cerebral perfusion. Yet, CTP which is deemed as a widely available diagnostic tool is able to provide quick and minimally invasive assessment for brain perfusion [32, 33]. Transcranial Doppler (TCD) is relatively inexpensive and widely available but does not provide additional information of the brain parenchyma and lack of appropriate transtemporal windows and poor cooperation, especially among the elderly [34]. Although no ideal or specific imaging modality is available for demonstration and accurate measurement of the collateral circulation [35], we used DSA, the gold standard for angiography, in our study to provide insight into collateral flow. A recent study has demonstrated the interrelation between the collateral circulation and cerebral perfusion, while the observational tool for collateral is relied on CTA [36]. However, the assessment of collateral filling by CTA depends largely on the timing of imaging, and delayed contrast enhancement of collateral vessels can lead to an underestimation of collateral blood supply.

Recent studies have suggested that baseline CBV impairment is associated with future ischemic events and patients with ICAO are approximately 4 times more likely to develop stroke or TIA [37]. However, in our study, no significant effects on CBV were found in regions of ipsilateral ICA. The reason may be that the blood flow velocity and vascular permeability of the involved artery stenosis are different from those of occluded artery. Compared with CBV, the TTP and MTT appear to be more sensitive to hemodynamic change since they directly track the traversal of contrast medium through cervical to the cerebral vascular circuit [38]. Furthermore, prolonged TTP and MTT are associated with delayed perfusion which would weaken the thromboemboli clearance ability and increase the risk of subsequent stroke [39]. Our findings revealed that rTTP and rMTT in CS patients with good collaterals (Grade 3) showed nonsignificant variations in selected ROIs compared with other collateral pathways. These results were in line with other previous conclusions that the CoW opening (grade 1 or grade 3) would not affect perfusion in the ipsilateral MCA territory in CS patients [10, 40, 41]. Besides, our study that the mean rCBF in selected ROIs revealed no difference in patients with various collateral circulation showed agreement with previous studies which were measured by TCD and MR angiography [42, 43].

RETRACTED

In our study, we found that the presence of collaterals in CS patients held strong relationship with the degree of stenosis and higher percentage of grades 2 or 3 was noticed in patients with carotid NO. Even though complete and fully functional CoW exists only in approximately 30% of elderly (arteriosclerotic) patients [44], these results still reached a consensus with some studies before using DSA and iFlow tool that reported more collateral recruits were related to higher degree of CS [21]. This can be highly explained from a hemodynamic perspective. An expected slightly lower blood pressure at the branching of MCA from ICA would lead to reduced blood flow rate (BFR) in ipsilateral MCA, inducing more cerebral flow to transmit from the contralateral side toward the ipsilateral side [45].

Conventionally, hemodynamically significant CS is described as a decrease in luminal diameter of a carotid artery by 70% to 80% [46]. Thus, degree of stenosis was used to stratify stroke risk in patients with CS in previous large, randomized trials [2]. Nonetheless, our study demonstrated that no significant relationship was noticed between the degree of stenosis and compromised flow status in temporal lobe and basil ganglia while frontal lobe showed significant elevation in the ratio of MTT and TTP, suggesting impaired perfusion in the frontal lobe beyond the severity of CS. The hypothesis of this phenomenon may be explained by cerebral blood flow redistribution owing to cerebral autoregulatory vasodilatation effects in patients with carotid NO. MCA territories which are responsible for more critical neurological functions would be guaranteed in priority when encountering insufficient CBF. However, reduction of MTT and TTP can influence regional or global frontal lobe function, contributing to impaired acquisition, execution, and complex decision-making [47, 48].

Moreover, according to the Spencer curve, the blood flow in ICA reduces nonlinearly with the degree of CS while drastically drops under a severe stenosis [49]. Hence, we further analyzed the patients with carotid NO who deemed to have extremely high risk of cerebral ischemia and strongly recommended to be revascularized. The results revealed that intact CoW may hold nonsignificant change to the perfusion of unilateral moderate CS while lead to significant reduction to the rMTT and rTTP values of hemicerebrum with ipsilateral carotid NO, suggesting that compensatory blood flow from contralateral ICA via anterior communicating artery (ACoA) would largely alleviate ipsilateral hypoperfusion and decrease the ischemia risk consequently. Jongen et al. [17] investigated the interrelation between the stenosis degree, configuration of collaterals, and cerebral perfusion. Specifically, cerebral perfusion parameters were related to increasing severity of CS while no correlation was found with the configuration of the CoW. Yet, our findings showed deviation on these results, indicating that linear hemodynamic compromise was barely related to stenosis degree in MCA territory while intact CoW played a pivotal role on perfusion parameters among NO patients. This discrepancy can be explained that patients enrolled in this subgroup were all defined as carotid NO and statistical bias would be decreased. Besides, according to our results, complete collateral circulation (grade 3) was noted in more patients with carotid NO and that was paramount for maintaining cerebral perfusion with ipsilateral severe CS and may further decline distal infarction risks. Similarly, Barnett and Meldrum [50] mentioned that the presence of hemodynamic compensation via CoW may be clinically useful to define intraoperative ischemia risk in CS patients. Our prior study also suggests that sufficient collateral circulation via CoW may promote ipsilateral cerebral perfusion and mitigate white matter change in patients with severe CS [51].

RETRACTED

The present study has some limitations. First, the small sample size and retrospective cross-sectional design limit the interpretation and generalizability of the study results. Secondly, another crucial point is the eyeball estimation of the collateral pathway to evaluate the hemodynamic compromise status relying on DSA images. This might lead to a certain subjectivity as no validated definition criteria for this method have been established. Thirdly, postoperative ischemic events are not evaluated to testify the influence of hemodynamic deficit, while this part would be further investigated in future studies. Finally, CTP is a widely available diagnostic tool. However, limited to expense, availability, and low spatial and temporal resolution, PET and single-photon emission tomography are not performed in our study which may hold more precise quantification of cerebral perfusion.

## 5. Conclusions

In conclusion, this study illustrates an effective assessment for collateral circulation based on DSA and its correlation with cerebral hemodynamic status in CS patients. Primarily, the grades of collateral circulation alone are hard to illuminate its significant correlation with ipsilateral cerebral perfusion and the severity of CS shows no linear relevance with hemodynamic deficit except for the frontal lobe. Secondly, complete collateral circulation is noticed in more patients with carotid NO and may serve as an objective angiographic parameter for assessing ipsilateral cerebral perfusion deficits among these patients. Finally, we initially hypothesize that the increased risk of stroke in CS patients is not only associated with degree of carotid stenosis and plaque stability but also collateral circulation. Hence, more dimensions need to be investigated in our future studies so as to make a better risk stratification and therapeutic strategy recommendations for CS patients.

RETRACTED

## Figures and Tables

**Figure 1:** DSA in patients with ipsilateral sided carotid stenosis showing collateral circulation from contralateral carotid artery injection. (a) Grade 1 indicates no or slight collateral distribution, often with dilution; (b) Grade 2 indicates small but definite collateral supply; (c) Grade 3 indicates near complete collateral with cross-filling of the ipsilateral middle cerebral artery after contralateral carotid injection; (d) illustrated the image of carotid NO: as grey arrow points, significant stenosis of ICA bifurcation with poor antegrade blood flow; (E) the grey arrows show the reduced diameter of the ICA without full collapse and delayed cranial arrival of ICA.

**Figure 2:** Relation between the degree of carotid stenosis and the collateral circulation grades. Chi-square test.  ^*∗*^*P* < 0.05; ^*∗∗*^*P* < 0.01; ^*∗∗∗*^*P* < 0.0001.

**Table 1:** Baseline characteristics of the study population (*n* = 124).

**Characteristics**	***N* (%)**
*Demographic characteristics*	
Age^1^, years	68.26 ± 8.36
Male	102 (82.25%)
Left side	68 (54.84%)
Previous stroke	18 (14.52%)
Aspirin	107 (86.29%)
Clopidogrel	86 (69.35%)
Warfarin	10 (8.06%)
*Preoperative degree of stenosis*	
50–70%	21 (16.94%)
70–90%	35 (28.23%)
Near-occlusion	68 (54.84%)
*Comorbidities*	
Ischemic heart disease	26 (20.97%)
Diabetes mellitus	32 (25.81%)
Hyperlipidemia	44 (35.48%)
Hypertension	91 (73.39%)
Tobacco abuse	49 (39.52%)
*Collateral circulation*	
Grade 1	74 (59.68%)
Grade 2	27 (21.77%)
Grade 3	23 (18.55%)

TIA: transient ischemia attack. Values denote numbers unless specified otherwise. ^1^Mean ± SD with range in parenthesis.

**Table 2:** Correlation between cerebral CTP parameters and collateral circulation in selected ROIs.

**ROIs**	**Grade 1**	**Grade 2**	**Grade 3**	*P * **value**
*rCBV*				
Frontal lobe	1.094 ± 0.378	1.122 ± 0.429	1.133 ± 0.512	0.926
Basal ganglia	1.061 ± 0.360	1.057 ± 0.413	1.052 ± 0.408	0.996
Temporal lobe	1.158 ± 0.450	1.077 ± 0.449	1.218 ± 0.528	0.533
Occipital lobe	1.065 ± 0.291	1.172 ± 0.520	1.047 ± 0.230	0.381
*rCBF*				
Frontal lobe	1.000 ± 0.334	1.113 ± 0.759	1.042 ± 0.241	0.621
Basal ganglia	1.006 ± 0.291	0.953 ± 0.291	1.038 ± 0.221	0.592
Temporal lobe	0.999 ± 0.295	0.839 ± 0.293	1.107 ± 0.441	0.344
Occipital lobe	1.033 ± 0.539	1.226 ± 0.894	1.122 ± 0.323	0.419
*rMTT*				
Frontal lobe	1.251 ± 1.005	1.299 ± 1.243	1.052 ± 0.375	0.720
Basal ganglia	1.114 ± 0.424	1.107 ± 0.382	1.055 ± 0.486	0.865
Temporal lobe	1.247 ± 0.570	1.178 ± 0.341	1.099 ± 0.419	0.514
Occipital lobe	1.122 ± 0.393	1.049 ± 0.393	1.037 ± 0.317	0.565
*rTTP*				
Frontal lobe	1.024 ± 0.075	1.045 ± 0.095	1.039 ± 0.085	0.959
Basal ganglia	1.024 ± 0.106	1.068 ± 0.251	1.004 ± 0.079	0.318
Temporal lobe	1.119 ± 0.271	1.059 ± 0.129	1.010 ± 0.085	0.058
Occipital lobe	1.058 ± 0.098	1.042 ± 0.076	1.018 ± 0.083	0.238

All data are means ± SE. Note: ROI: region of interest; rCBV: relative cerebral blood volume; rCBF: relative cerebral blood flow; rMTT: relative mean transit time; rTTP: relative time to peak.  ^*∗*^*P* < 0.05.

RETRACTED

**Table 3:** Correlation between degree of carotid stenosis and collateral circulation.

**Collateral circulation**	**50–70%, *n*** **=** **21**	**70–90%, *n*** **=** **35**	**Near-occlusion, *n*** **=** **68**	*P * **value**
Grade 1	19 (90.48%)	25 (71.43%)	24 (35.29%)	<0.0001^*∗∗∗∗*^
Grade 2	1 (4.76%)	7 (20.00%)	22 (32.35%)	
Grade 3	1 (4.76%)	3 (8.57%)	22 (32.35%)	

Note: chi-square test.  ^*∗*^*P* < 0.05; ^*∗∗*^*P* < 0.01; ^*∗∗∗∗*^*P* < 0.0001.

**Table 4:** Correlation between cerebral CTP parameters and degree of carotid stenosis in selected ROIs.

**ROIs**	**50–70%**	**70–90%**	**Near-occlusion**	*P * **value**
*rMTT*				
Frontal lobe	1.033 ± 0.152	1.090 ± 0.292	1.235 ± 0.291	0.037^∗^
Basal ganglia	1.027 ± 0.382	1.084 ± 0.342	1.144 ± 0.308	0.255
Temporal lobe	1.035 ± 0.422	1.374 ± 0.513	1.362 ± 0.919	0.331
*rTTP*				
Frontal lobe	0.994 ± 0.070	1.021 ± 0.076	1.054 ± 0.084	0.026^∗^
Basal ganglia	0.981 ± 0.075	1.048 ± 0.137	1.034 ± 0.072	0.065
Temporal lobe	0.994 ± 0.099	1.018 ± 0.059	1.044 ± 0.076	0.158

All data are means ± SE. Note: ROIs: regions of interest; rMTT: relative mean transit time; rTTP: relative time to peak.  ^*∗*^*P* < 0.05.

**Table 5:** Comparison between cerebral perfusion and collateral circulation in patients with carotid near-occlusion.

**ROIs**	**Grade 1**	**Grade 2**	**Grade 3**	*P * **value**
*Frontal lobe*				
rCBF	1.09 ± 0.34	0.95 ± 0.25	1.00 ± 0.28	0.349
rMTT	1.07 ± 0.38	0.99 ± 0.26	1.03 ± 0.29	0.729
rTTP	1.07 ± 0.22	1.06 ± 0.13	1.05 ± 0.24	0.917
*Basal ganglia*				
rCBF	0.90 ± 0.22	0.95 ± 0.28	1.01 ± 0.25	0.322
rMTT	1.21 ± 0.28	1.07 ± 0.29	0.96 ± 0.29	0.024^∗^
rTTP	1.13 ± 0.15	1.06 ± 0.13	1.02 ± 0.13	0.040^∗^
*Temporal lobe*				
rCBF	1.08 ± 0.25	1.02 ± 0.23	0.99 ± 0.24	0.449
rMTT	1.08 ± 0.21	1.03 ± 0.20	1.02 ± 0.16	0.525
rTTP	1.10 ± 0.10	1.05 ± 0.09	1.03 ± 0.08	0.047^∗^

All data are means ± SE. Note: ROIs: regions of interest; rCBF: relative cerebral blood flow; rMTT: relative mean transit time; rTTP: relative time to peak.  ^*∗*^*P* < 0.05.

RETRACTED

## Data Availability

The simulation experiment data used to support the findings of this study are available from the corresponding author upon request.

## Abbreviations

CS: Carotid stenosis
CTP: Computed tomography perfusion
CEA: Carotid endarterectomy
DSA: Digital substruction angiography
MCA: Middle cerebral artery
NO: Near-occlusion
CCA: Common carotid artery
ICA: Internal carotid artery
ICAO: Internal carotid artery occlusion
VA: Vertebral artery
CBV: Cerebral blood volume
CBF: Cerebral blood flow
MTT: Mean transit time
TTP: Time to peak
ROIs: Regions of interest
CoW: Circle of Willis
CTA: Computed tomography angiography
TCD: Transcranial Doppler
ASL: Arterial spin labeling
MRI: Magnetic resonance imaging
TIA: Transient ischemic attack
BFR: Blood flow rate
ACoA: Anterior communicating artery
PET: Positron emission tomography.
